# Analysis of Distributions of HPV Infection in Females with Cervical Lesions in the Western District of Beijing Chaoyang Hospital

**DOI:** 10.1155/2022/5422748

**Published:** 2022-03-14

**Authors:** Meili Gong, Chen Chen, Huirong Zhao, Liyuan Guo, Mingxia Sun, Meiyu Song

**Affiliations:** Department of Obstetrics and Gynecology, Beijing Chaoyang Hospital Affiliated to Capital Medical University, Beijing, China

## Abstract

**Objective:**

To analyze the distribution of human papilloma virus (HPV) infection in women with cervical lesions of different grades and analyze the relationship of high-risk HPV and cervical lesions in order to facilitate targeted prevention.

**Methods:**

The infection status of HPV subtype was statistically analyzed in patients who underwent colposcopy examination from April 2017 to June 2019.

**Results:**

The infection rate of HPV was 81.4% in chronic cervicitis, 82.9% in 1ow-grade squamous intraepithelial lesion (LSIL), 63.7% in HSIL (high-grade squamous intraepithelial lesion), and 50% in cervical squamous cell carcinoma (CSCC). Among the 16 high-risk HPV types, the top six HPV types with the comprehensive infection rates were HPV16 > HPV52 > HPV58 > HPV18 > HPV51 > HPV53 in turn, and the infection rates were 23.3%, 14.8%, 13.3%, 9.8%, 9.2%, and 8.8%, respectively. The infection rates of HPV16 in chronic cervicitis group, LSIL group, and HSIL group were significantly different. There was no significant difference in the injection rates of HPV52, HPV58, and HPV18 among the three groups. HPV infection rates were highest in the 31–40 years old group, followed by the 41–50 years old group.

**Conclusion:**

The distribution of different types of HPV varies in different tissue types, which can be used to develop relevant vaccines to achieve better prevention and treatment of cervical cancer.

## 1. Introduction

Cervical cancer, one of the most common gynecological malignancies, is the fourth most common cancer among women. In 2018, there were an estimated 570,000 new cases globally, accounting for 6.6% of all female cancers [1]. The number of new cases of cervical cancer in China is increasing at a rate of 15,000 per year, ranking the second in the world [2]. Human papilloma virus (HPV) infection is a high-risk factor leading to cervical cancer, which seriously affects women's physical and mental health and reproductive outcomes [3]. The occurrence of cervical squamous intraepithelial lesion (SIL) and cervical cancer is mainly related to the persistent high-risk HPV infection. More than 30 types of HPV are now known to be associated with reproductive tract infections. Low-risk HPV6 and 11 are most common in genital warts. High-risk HPV is the type associated with genital cancers, especially cervical cancer. HPV16 and 18 infections account for 70% of cervical cancer, while the other 12 high-risk HPV types (31, 33, 35, 39, 45, 51, 52, 56, 58, 59, 68, and 73) account for 1–9% of cervical cancer [4]. This article analyzed the distribution of different types of HPV in different tissue types of cervical lesions, which played an important role in the prevention, diagnosis, and treatment of cervical cancer.

In this paper, we analyzed the HPV subtype infection of 1259 patients with cervical lesions, and the correlation between high-risk HPV infection and cervical lesions, so as to provide targeted prevention, diagnosis, and treatment for cervical cancer.

## 2. Materials and Methods

### 2.1. General Information

A total of 1259 patients who underwent the colposcopy clinic in Beijing Cahoyang Hospital Affiliated to Capital Medical University from April 2017 to June 2019 were selected, aged 18–80 years old, with an average of 41.48 ± 10.71 years old. Among them, 108 cases were HPV-negative, and 1,151 cases were HPV infection. The study was approved by the Ethic Committee of Beijing Chaoyang Hospital Affiliated to Capital Medical University.

Inclusion criteria: patients with abnormal cervical TCT or high-risk HPV infection require further colposcopy examination. Exclusive criteria: (1) patients without performed HPV typing test; (2) patients with genital tract malformation; and (3) patients with severe genital tract infections.

### 2.2. Specimen Sampling

The patients presented with a cystolithotomy position to fully expose the cervix. The special cervical detection brush was placed inside the cervical canal and rotated clockwise for 5 times. The cervical brush was put into a special tube and sent to the laboratory for testing.

### 2.3. Cervical Thin Prep Liquid-Based Cytology Test (TCT) and Pathological Examination

Cervical cells in fluid-based thin layer were detected by the new Berberian TCT test, and TBS (2001) classification was used for cytological diagnosis. TBS classification standard: atypical squamous cells (ASC), negative for intraepithelial lesion or malignancy (NIM), 1ow-grade squamous intraepithelial lesion (LSIL), and high-grade squamous intraepithelial lesion (HSIL). The pathological diagnosis of cervical squamous epithelial lesions was divided into LSIL and HSIL by WHO classification (2014).

### 2.4. HPV Types Detection

The HPV types were detected by the HPV typing test kit of Cape Company, and according to the reagent instruction, 27 genotypes of human HPV can be identified, including high-risk HPV: 16, 18, 31, 33, 35, 39, 45, 51, 52, 53, 56, 58, 59, 66, 68, and 82 and low-risk HPV: 42, 44, 81, etc.

### 2.5. Statistical Analysis

SPSS 22.0 system software was used for data analysis. The infection rates of different types of HPV in different groups were analyzed by *χ*^2^ test. Fisher test was used when the number of cases was less than 5. *p* < 0.05 was considered statistically significant.

## 3. Results

### 3.1. Comparison of HPV Infection Rates among Different Cervical Lesions

Among 1259 patients, LSIL was the most common pathological diagnosis, followed by chronic cervicitis and HSIL, and cervical squamous cell carcinoma (CSCC) was the least (Table 1). The HPV infection rate was 81.4% among 221 patients with chronic cervicitis, 82.9% among 847 patients with LSIL, 63.7% among 179 patients with HSIL, and 50% among 12 patients with CSCC (Table 1). There was significant difference in HPV infection rate among the four groups (*χ*^2^ = 40.447, *p* < 0.01). Pairwise comparison showed that there was significant difference in HPV infection rate between HSIL and LSIL group (*χ*^2^ = 33.442, *p* < 0.01), HSIL and chronic cervicitis group (*χ*^2^ = 16.017, *p* < 0.01), chronic cervicitis and CSCC group (*χ*^2^ = 5.174, *p*=0.017), and LSIL and CSCC group (*χ*^2^ = 6.706, *p* < 0.01). There was no notable difference in HPV infection rate between chronic cervicitis and LSIL group (*χ*^2^ = 0.250, *p* > 0.05) and HSIL and CSCC group (*χ*^2^ = 0.411, *p* > 0.05).

### 3.2. Comparison of Single and Multiple HPV Infections in Different Cervical Lesions

Single HPV infection accounted for 67.8% in the chronic cervicitis group, 60.7% in the LSIL group, 57.9% in the HSIL group, and 66.7% in CSCC group (Table 2). In general, single HPV infection accounted for 61.7%. There was no significant difference between single infection and multiple infection among the four groups (*χ*^2^ = 3.94, *p*=0.268). There was no significant difference in infection rate between single and multiple infections between chronic cervicitis and LSIL group (*χ*^2^ = 3.064, *p*=0.085), HSIL and LSIL group (*χ*^2^ = 0.319, *p*=0.321), HSIL and chronic cervicitis group (*χ*^2^ = 2.957, *p*=0.056), HSIL and CSCC group (*χ*^2^ = 0.185, *p*=0.509), chronic cervicitis and CSCC group (*χ*^2^ = 0.003, *p*=0.631), and LSIL and CSCC group (*χ*^2^ = 0.091, *p*=0.56).

### 3.3. Distribution of HPV Subtypes in Different Cervical Lesions

Among the 16 high-risk HPV subtypes, the HPV subtypes in the top six were HPV16 (23.3%), HPV52 (14.8%), HPV58 (13.3%), HPV18 (9.8%), HPV51 (9.2%), and HPV53 (8.8%) in descending order (Table 3). In the chronic cervicitis group, the top 6 subtypes of HPV infection rate were HPV58, HPV16, HPV51, HPV39, HPV52, and HPV18. In the LSIL group, the top 6 subtypes of HPV infection rates were HPV16, HPV52, HPV58, HPV18, HPV53, and HPV51. In HSIL group, the top 6 of subtypes of HPV infection rates were HPV16, HPV52, HPV18, HPV33, HPV58, and HPV53(51). In CSCC group, the subtypes of HPV infection rates were HPV16, HPV58, HPV18, and HPV68 (Table 3).

The infection rates of first 4 high-risk HPV subtypes in chronic cervicitis, LSIL, and HSIL group were compared and analyzed. The infection rate of HPV16 was significantly different in chronic cervicitis, LSIL, and HSIL group (*p* < 0.05, Table 4), while there were no differences in the infection rates of HPV52, HPV58, and HPV18 in the three groups (*p* > 0.05, Table 4).

### 3.4. HPV Infection in Cervical Lesions in Different Age Groups

Patients were divided into 6 groups according to age: ≤20 years old, 21–30 years old, 31–40 years old, 41–50 years old, 51–60 years old, and ≥61 years old. The group with the highest HPV-positive infection rate was 31–40 years old, followed by 41–50 years old, and 51–60 years old (Table 5).

There was significant difference in age group of chronic cervicitis group (*χ*^2^ = 17.045, *p*=0.002, Table 6), while there was no significant difference in the age of HPV infection in the LSIL, HSIL, and CSCC groups (Table 6).

## 4. Discussion

HPV is closely related to cervical lesions and the occurrence and development of cervical cancer [5]. Studies have shown that almost all patients with cervical cancer are infected with HPV, and infections of HPV 6, 11, 16, 18, 31, 33, 45, 52, and 58 cause 90% of cervical cancer [6]. However, this study showed that the HPV infection rate of cervical cancer was 50%, which may be related to the small sample size and too much necrotic tissues of cervical cancer. Our study gives a clinical warning that cervical cancer cannot be completely ruled out, even of HPV is negative. It is necessary to make a comprehensive judgment combining with clinical symptoms and signs. Wu et al. discussed the role of FAMl9A4 gene methylation in the diagnosis of hrHPV-negative cervical cancer, which was considered to be related to epigenetic variation [7].

Qiu et al. [8] studied 263 patients with cervical cancer and found no statistically significant difference in HPV infection rates among CINI, II, III, and stage IV cervical cancer. This work showed that the HPV infection rate in LSIL was 82.9% and in HSIL was 63.75, and there were significant differences in the HPV infection rate between the four groups. However, there was no significant difference in HPV infection rate between chronic cervicitis and LSIL or HSIL and CSCC group. Therefore, there was a significant difference in HPV infection rate between the observation group (chronic cervicitis and LSIL) and the treatment group (HSIL and CSCC). Talia Malagon et al. found that the largest difference in HPV viral load occurred in normal and CIN1 type women, while the difference in viral load between CIN grades was small [9]. It was considered to be related to HPV infection type, infection time, HPV clearance time, and other factors. However, whether there is a trigger point between HPV infection and cervical grading lesions and its specific mechanism requires further study.

In the current work, the single high-risk HPV infection rate was higher than the multiple infection rate, indicating that the high-risk HPV infection was mainly single infection, which is basically similar to the single infection rate of HPV in other gynecological clinics [10]. There is still a great deal of controversy about whether multiple HPV infections promote further cervical lesions. Some scholars believe that multiple HPV infections may be related to the development of cervical abnormalities [11]. Even multiple HPV genotypes are related to the poor survival rate of cervical cancer [12]. Studies have also pointed out that patients with multiple infection of HPV do not significantly increase the risk of cervical cancer and cervical CIN compared with single infection [13]. Wu et al. [14] believed that coinfection of HPV16/18 with other hrHPVs was a common phenomenon, and single HPV16 infection had a higher risk of CIN3 progression. Li et al. [15] also found that the incidence of CIN2 in patients with single HPV16 infection was higher than that in patients with multiple HPV16 infection. However, our study showed that there was no significant difference between single and multiple HPV infection rates among different cervical lesions.

The genotypes of HPV infection are different in different regions and ethnic groups. The main high-risk HPV types in Mongolia are HPV16, 52, 58, 33, and 31, HPV16, 18, 52, and 58 in Japan, and HPV16, 58, 33, and 52 in South Korea [16]. There are also some differences in HPV infection among women of different regions and different economic levels in China [17]. Our study suggested that HPV infections were predominantly HPV16, 52, 58, 18, and 51. The current HPV nine-valent vaccine (anti-HPV6, 11, 16, 18, 31, 33, 45, 52, and 58 subtypes) has included the four HPVs with the highest infection. Therefore, according to the epidemiology of regional HPV, vaccines more suitable for inhibiting high-risk HPV subtypes in corresponding regions can be developed, so as to make the cervical cancer vaccine more accurate.

It has been reported that age is a factor influencing HPV infection and cervical lesions, and there are two peaks of HPV infection among women aged 20–30 years and 50–60 years [18]. Li et al. observed that HPV distribution in the whole age was U-shaped bimodal curve, with the highest HPV infection rate at <20 years old, and the second peak at >50 years old [19]. Our study indicated that the group with the highest HPV-positive infection rate was 31–40 years old, followed by 41–50 years old and 51–60 years old. However, there was no significant difference in the age of HPV infection in LSIL, HSIL, and CSCC groups. The findings may be associated with sexual activity and the large base of HPV screening population in this age group.

Previous study confirmed that the single baseline HPV test is a strong predictor of cervical abnormalities for a risk prediction model for cervical cancer [20]. However, the limitations of this study are that the sample size is small and the survey is based on a single hospital, and the information of patients' sexual behavior, number of sexual partners, lifestyle, and social and economic status are not collected. Therefore, there are insufficient practical guidelines for preventing HPV infection in high-risk group, and large prospective studies are needed to develop, screen, and validate risk prediction models.

## 5. Conclusion

In conclusion, we analyzed distribution of HPV infection in women with different grades of cervical lesions and the relationship between high-risk HPV and cervical lesions, providing a basis for the future targeted development of cervical cancer vaccine. It is also of great significance to evaluate the effectiveness by establishing a model to warn the disease progression and reduce psychological anxiety, examination times, and cost of patients with HPV infection.

## Figures and Tables

**Table 1:** HPV infection in different cervical lesions (case (%)).

	*n*	HPV-negative	HPV-positive					
			1	2	3	4	≥5	Total
Cervicitis	221	41 (18.6)	122 (55.2)	51 (23.1)	7 (3.2)	0	0	180 (81.4)
LSIL	847	145 (17.1)	426 (50.3)	216 (25.5)	49 (5.8)	6 (0.7)	5 (0.6)	702 (82.9)
HSIL	179	65 (36.3)	66 (36.8)	35 (19.6)	11 (6.1)	2 (1.1)	0	114 (63.7)
CSCC	12	6 (50)	4 (33.3)	2 (16.7)	0	0	0	6 (50)

**Table 2:** HPV single and multiple infection data (case (%)).

	Single	Multiple	Total
Cervicitis	122 (67.8)	58 (32.2)	180
LSIL	426 (60.7)	276 (39.3)	702
HSIL	66 (57.9)	48 (42.1)	114
CSCC	4 (66.7)	2 (33.3)	6
Total	618 (61.7)	384 (38.3)	1002

**Table 3:** The case and proportion of HPV subtype infection.

HPV	HPV-positive	Cervicitis (*n* = 221)	LSIL (*n* = 847)	HSIL (*n* = 179)	CSCC (*n* = 12)
HPV16	293 (23.3)	29 (13.1)	174 (20.5)	83 (46.4)	7 (58.3)
HPV18	124 (9.8)	22 (10.0)	81 (9.6)	20 (11.1)	1 (8.3)
HPV31	53 (4.2)	6 (2.7)	41 (4.8)	6 (3.3)	0
HPV33	61 (4.8)	6 (2.7)	35 (4.1)	20 (11.1)	0
HPV35	21 (1.7)	3 (1.4)	15 (1.8)	3 (1.7)	0
HPV39	95 (7.5)	24 (10.9)	68 (8.0)	3 (1.7)	0
HPV45	8 (0.6)	1 (0.5)	7 (0.8)	0	0
HPV51	116 (9.2)	28 (12.7)	75 (8.9)	13 (7.3)	0
HPV52	186 (14.8)	23 (10.4)	136 (16.1)	27 (15.0)	0
HPV53	111 (8.8)	22 (10.0)	76 (9.0)	13 (7.3)	0
HPV56	71 (5.6)	11 (5.0)	52 (6.1)	8 (4.5)	0
HPV58	36 (13.3)	30 (13.6)	116 (13.7)	19 (10.6)	2 (16.7)
HPV59	36 (2.9)	6 (2.7)	27 (3.2)	3 (1.7)	0
HPV66	63 (5.0)	8 (3.6)	44 (5.2)	11 (6.1)	0
HPV68	37 (2.9)	9 (4.1)	24 (2.8)	3 (1.7)	1 (8.3)
HPV81	27 (2.1)	2 (0.9)	23 (2.7)	2 (1.1)	0
HPV82	4 (0.3)	1 (0.5)	2 (0.2)	1 (0.6)	0
HPV42	9 (0.7)	1 (0.5)	7 (0.8)	1 (0.5)	0
HPV44	7 (0.6)	1 (0.5)	6 (0.7)	0	0
HPV-negative	108 (8.6)	22 (10.0)	74 (8.7)	9 (5.0)	3 (25.0)

**Table 4:** Distribution of HPV16, 52, 58, and 18 in different cervical lesions (case (%)).

	*n*	HPV16	HPV52	HPV58	HPV18
Cervicitis	221	299 (13.1)	23 (10.4)	30 (13.6)	22 (10.0)
LSIL	847	174 (20.5)	136 (16.1)	116 (13.7)	81 (10.0)
HSIL	179	83 (46.4)	27 (15.1)	19 (10.6)	20 (11.2)
*χ* ^2^		70.395	4.412	1.249	0.433
*p*		0.000	0.093	0.535	0.805
LSIL and HSIL	*χ* ^2^	52.496	0.105	1.227	0.432
	*p*	0.000	0.746	0.268	0.296
Cervicitis and LSIL	*χ* ^2^	6.270	4.415	0.002	0.031
	*p*	0.012	0.036	0.531	0.473
Cervicitis and HSIL	*χ* ^2^	54.224	1.978	0.806	0.156
	*p*	0.000	0.16	0.229	0.407

**Table 5:** The case of HPV-positive grouped by age.

Age	HPV-positive	HPV16	HPV52	HPV58	HPV18	HPV51	HPV53
≤20	4(0.3)	3	0	0	0	1	0
21–30	185(14.7)	46	30	31	16	20	11
31–40	468(37.2)	119	63	60	56	35	45
41–50	307(24.4)	65	52	40	26	33	22
51–60	240(19.1)	43	36	30	22	24	26
≥61	55(4.4)	17	5	6	4	3	7

**Table 6:** The positive case of age-specific HPV infection in different cervical lesions.

Age	LSIL	HSIL	Cervicitis	CSCC
21–30	114	32	35	0
31–40	310	77	78	3
41–50	198	38	68	3
51–60	180	22	33	5
≥61	43	8	3	1
*χ* ^2^	0.642	1.4	17.045	4.673
*p*	0.958	0.393	0.002	0.179

## Data Availability

The datasets used and/or analyzed during the current study are available from the corresponding author on reasonable request.
